The article "Chicory (Cichorium intybus L.) Root Extract Regulates the Oxidative Status and Antioxidant Gene Transcripts in CCl4-Induced Hepatotoxicity" was retracted in 2017. Reasons: manipulated images; results that could not be reproduced; duplicated images; duplicated data.

# Chicory (*Cichorium intybus* L.) Root Extract Regulates the Oxidative Status and Antioxidant Gene Transcripts in CCl_4_-Induced Hepatotoxicity

**DOI:** 10.1371/journal.pone.0121549

**Published:** 2015-03-25

**Authors:** Yasser S. El-Sayed, Mohamed A. Lebda, Mohammed Hassinin, Saad A. Neoman

**Affiliations:** 1 Department of Veterinary Forensic Medicine and Toxicology, Faculty of Veterinary Medicine, Damanhour University, Damanhour, Egypt; 2 Department of Biochemistry, Faculty of Veterinary Medicine, Alexandria University, Edfina, Egypt; 3 Department of Clinical Biochemistry, College of Medicine, King Abdulaziz University Jeddah, Jeddah, Saudi Arabia; 4 Department of Medical Biochemistry, Faculty of Medicine, Tanta University, Tanta, Egypt; Universidad Pablo de Olavide, Centro Andaluz de Biología del Desarrollo-CSIC, SPAIN

## Abstract

The ability of *Cichorium intybus* root extract (chicory extract) to protect against carbon tetrachloride (CCl_4_)-induced oxidative stress and hepatotoxicity was evaluated in male rats. The rats were divided into four groups according to treatment: saline (control); chicory extract (100 mg/kg body weight daily, given orally for 2 weeks); CCl_4_ (1 ml/kg body weight by intraperitoneal injection for 2 consecutive days only); or chicory extract (100 mg/kg body weight daily for 2 weeks) + CCl_4_ injection on days 16 and 17. The levels of hepatic lipid peroxidation, antioxidants, and molecular biomarkers were estimated twenty-four hours after the last CCl_4_ injection. Pretreatment with chicory extract significantly reduced CCl_4_-induced elevation of malondialdehyde levels and nearly normalized levels of glutathione and activity of glutathione S-transferase, glutathione peroxidase (GPx), glutathione reductase, catalase (CAT), paraoxonase-1 (PON1), and arylesterase in the liver. Chicory extract also attenuated CCl_4_-induced downregulation of hepatic mRNA expression levels of *GPx1*, *CAT* and *PON1* genes. Results of DNA fragmentation support the ability of chicory extract to ameliorate CCl_4_-induced liver toxicity. Taken together, our results demonstrate that chicory extract is rich in natural antioxidants and able to attenuate CCl_4_-induced hepatocellular injury, likely by scavenging reactive free radicals, boosting the endogenous antioxidant defense system, and overexpressing genes encoding antioxidant enzymes.

## Introduction

The liver is a vital organ that plays a central role in transforming and clearing chemicals and is susceptible to the toxicity from these agents [1]; therefore it is an important target organ of the toxicity of drugs, xenobiotics, and oxidative stress [2]. Hepatotoxicity is presently the most widespread pathology worldwide, representing up to 83% of all cases and the most serious health problems [3]. Free radicals and reactive oxygen species are increasingly believed to play a crucial role in the initiation and progression of liver diseases, independent of the original causal agent [4]. Carbon tetrachloride (CCl_4_) is a selective hepatotoxic chemical agent that is metabolized by the cytochrome P450 into highly reactive metabolites including trichloromethyl free radical (CCl_3_^•^) and trichloromethylperoxy radical (CCl_3_O_2_^•^). In turn, the generated free radicals decrease antioxidant enzymes activity and cause membrane lipid peroxidation [5]. Free radicals of CCl_4_ reduce glutathione (GSH) of phase II detoxification enzymes and GSH-dependent antioxidant enzymes, and considered substrates to induce oxidative stress, which is an important factor in acute and chronic hepatic injuries [6–8]. The depletion of these antioxidant enzymes occurs as consequences of the controlling action towards peroxy radicals generated by CCl_4_. Moreover, ROS cause oxidative DNA damage [9]. Therefore, the use of antioxidants play a significant role as antihepatotoxic potential by eliminating ROS and free radicals, and neutralizing lipid peroxides.

Recently, an interest is increasing in the use of herbal medicine for protection and/or therapies of hepatic disorders [10]. Chicory (*Cichorium intybus*), a member of the Asteraceae family, is a well-known herb possessing various biological activities. It was grown by ancient Egyptians as a medicinal plant, vegetable crop, and animal feed [11]. Chicory is native to Europe and Asia and has been widely used in traditional therapy for the medication gastrointestinal and inflammatory disorders [12]. Important phytochemicals are distributed throughout the plant; however, the primary contents are present in the root. Fresh chicory root typically is well characterized [12, 13]. Extracts of chicory root have been stated to have antimicrobial [14–16], antihyperglycemic [17, 18], immunostimulant [19, 20], antitoxic [21–23], antiinflammatory [24], and tumor-inhibitory activities [25, 26]. We thus evaluated the hepatoprotective and antioxidant potentials of an aqueous chicory root extract (CE) on CCl_4_-induced acute hepatic injury by elucidating the biochemical and molecular mechanisms, as well as the DNA damage underlying these effects.

## Materials and Methods

### Ethics statement

All experiments were performed in accordance with Animal Research: Reporting *In Vivo* Experiments guidelines for the care and use of laboratory animals [27] and were approved by Animal Care Review Committee of the Faculty of Medicine, Tanta University, Tanta, Egypt (Ethical Issue No: AS223587/2014). The animals received humane care according to the “Guide for the Care and Use of Laboratory Animals” of the United State National Academy of Sciences, and all efforts were made to minimize their suffering.

### Chemicals

CCl_4_ (CAS Number 56–23–5) was obtained from Sigma-Aldrich Co. Co. (St. Louis, MO, USA). All other chemicals were reagent grade and were commercially available from local distributors in Egypt. Assay kits for the measurement of malondialdehyde (MDA), reduced glutathione (GSH), glutathione S-transferase (GST), glutathione peroxidase (GPx), glutathione reductase (GR), and catalase (CAT) were purchased from Biodiagnostic Co. (Cairo, Egypt). QuantiFast SYBR Green PCR Kit was obtained from QIAGEN GmbH (Hilden, Germany), and the GoScript Reverse Transcription System was obtained from Promega (Madison, WI, USA).

### Plant material and extraction

The roots of *C*. *intybus* L. were collected from a local market for herbs and medicinal plants. Staff members of the Botany Department, Faculty of Agriculture, Alexandria University, Alexandria, Egypt authenticated the identity of the plants. The roots were washed, dried and ground to a coarse consistency. After that, the powder was passed through a mesh (particle size: 40 mm) and stored in an airtight container at room temperature. The powdered material was extracted with water through a simple maceration procedure at room temperature for 7 days in a conical flask with continuous shaking and stirring. The extract was filtered and dried by evaporation in a hot air oven at 50°C, with a percentage yield of 16% *w*/*w*. The aqueous extracts were formulated as suspensions in distilled water containing few drops of Tween 80 [28]. The strength of the suspension depended on the dose administered and was expressed as the weight of the dried extract.

### Phytochemical screening of the extract

Total phenolic content of the CE was assessed using the Folin—Ciocalteu method [29]. The blue color formed after the oxidation of the Folin—Ciocalteu reagent with the extract was measured at 760 nm against a blank reagent. Total phenolic content was calculated from the gallic acid calibration curve. Additionally, phytochemical tests were performed on CE for the assessment of other active constituents including; alkaloids, flavonoids, tannins, saponins, anthraquinones, steroids and terpenoids [30, 31].

### Animals and treatments

Male Sprague—Dawley rats (10 weeks old, approximately 200–250 g) were obtained from the animal breeding unit at the Medical Research Institute, Alexandria University, Egypt. The rats were housed in a room at a controlled temperature (23 ± 1°C) and humidity (55 ± 5%), with a 12 h dark/light cycle and *ad libitum* access to food and water. All rats were acclimatized in metal cages for one week prior to the experiment to ensure normal growth and behavior. After the acclimatization period, the rats were randomly divided into four groups of ten animals each. Group I, the control group, received an intraperitoneal (i.p) injection of 1 ml/kg body weight (bwt) saline on two consecutive days. Group II received 100 mg/kg bwt CE orally for two weeks. Group III received an i.p injection of 1 ml/kg bwt CCl_4_/olive oil (1:1 *v*/*v*) on two consecutive days. Group IV received 100 mg/kg bwt CE orally for two weeks and i.p injections of 1 ml/kg bwt CCl_4_/olive oil (1:1 *v*/*v*) on days 16 and 17. Twenty-four hours after the second CCl_4_ injection, the rats were decapitated, and their livers were carefully dissected and cleaned of extraneous tissues and stored at −70°C for biochemical, molecular, and genetic analysis.

### Measurement of tissue lipid peroxidation and antioxidant markers

To evaluate lipid peroxidation and antioxidant status in the liver, tissue samples were homogenized individually in 0.1 M phosphate buffer (pH 7.4), then centrifuged at 14,000 ×g for 15 min at −4°C. Aliquots of the supernatant were utilized for the spectrophotometric estimation of tissue MDA and GSH levels, as well as the activities of GST, GPx, CAT, GR, paraoxonase 1 (PON1) and arylesterase (AE) enzymes. Lipid peroxides measured as the MDA concentration were analyzed after the reaction with thiobarbituric acid in acidic medium at 95°C for 30 min to form thiobarbituric acid-reactive substances [32]. Absorbance of the resulting pink product was measured at 534 nm. The GSH assay was based on the reductive cleavage of 5, 5′-dithiobis (2-nitrobenzoic acid) by a sulfhydryl group to yield a yellow compound [33]. The amount of reduced chromogen (absorbance measured at 405 nm) is directly proportional to the GSH concentration. The GST assay was based on the conjugation of 1-chloro-2,4-dinitrobenzene with GSH [34]. Enzyme activity of GPx was determined by measuring oxidized glutathione, which is produced by the reduction of organic peroxide [35]. The GR assay was based on the method described by Goldberg and Spooner [36]. Briefly, 1 ml of 2.728 mM oxidized glutathione and 40 μl of liver homogenate were incubated for 5 min at 37°C. After incubation, the reaction was initiated by the addition of 200 μl of 1.054 mM NADPH. The decrease in absorbance was measured at 340 nm and recorded every 30 s for 5 min. The CAT activity was measured according to the method described by Aebi [37], in which CAT reacts with a known quantity of H_2_O_2_, and the reaction was stopped after 1 min with a CAT inhibitor. The remaining H_2_O_2_, in the presence of peroxidase, reacts with 3,5-dichloro-2-hydroxybenzene sulfonic acid and 4-aminophenazone to form a chromophore, with a color intensity that was inversely proportional to the amount of CAT in the sample. PON1 activity toward paraoxon (*O*,*O*-diethyl-O-*p*-nitrophenyl phosphate) was determined by measuring the initial rate of substrate hydrolysis to *p*-nitrophenol, whose absorbance was monitored at 405 nm in the assay mixture [38]. AE activity was determined as PON1 activity toward phenylacetate by measuring the initial rate of substrate hydrolysis to phenol, whose absorbance was monitored at 270 nm in the assay mixture [38]. Protein content in the liver homogenate was measured using bovine serum albumin as a standard.

### Reverse transcription-quantitative PCR (RT-qPCR)

Approximately 1 g of each liver sample was added immediately after dissection to 1 ml of TRIzol reagent (Invitrogen, Carlsbad, CA, USA) and homogenized using a Tissue Ruptor homogenizer (QIAGEN, GmbH, Germany). One milliliter of the tissue homogenate was transferred to a microfuge tube, and the total RNA was extracted by adding 0.2 ml chloroform. Next, the samples were vigorously vortexed for 15 s and incubated at room temperature for 3 min. After centrifugation at 12,000 ×*g* for 15 min at 4°C, the aqueous phase containing RNA was transferred to new tubes. The RNA was precipitated by mixing the aqueous phase with 0.5 ml isopropyl alcohol and incubating at room temperature for 10 min. After centrifugation at 12,000 ×*g* for 10 min at 4°C, the RNA pellets were washed by mixing and vortexing with 1 ml 75% ethanol. After centrifugation at 7,500 ×*g* for 5 min at 4°C, the RNA pellets were re-suspended in nuclease-free water (Life Technologies, Carlsbad, CA, USA). RNA concentration and purity were estimated from the optical density at 260 and 280 nm, respectively. The cDNA was prepared from 2 μg of total RNA using a Reverse Transcription System Kit (Promega) and a Bio-Rad Thermal Cycler (T100, Foster City, CA, USA). Briefly, the total RNA was activated at 70°C for 10 min, and a 20 μl reaction mix was created using 4 μl MgCl_2_, 2 μl of reverse transcription 10× buffer, 2 μl of 10 mM *d*NTP mixture, 0.5 μl of random primers, 0.75 μl of AMV reverse transcriptase enzyme, 1 ng RNA and nuclease-free water to a final volume of 20 μl. Then, the reaction was incubated at 42°C for 60 min followed by incubation at 94°C for 5 min. The cDNA was diluted up to 100 μl with nuclease-free water for PCR amplification. The RT-qPCR was performed using a QuantiFast SYBR Green PCR Master Mix kit (QIAGEN), and specific primers for the following antioxidant enzymes-related genes: *GPx*1, *CAT* and *PON*1 (Table 1). Each 25-μl reaction contained 12.5 μl of master mix, 2 μl of forward primer (10 pmol), 2 μl of reverse primer (10 pmol), 2 μl of cDNA, and 6.5 μl of nuclease-free water. The cycling parameters were: initial incubation at 95°C for 15 min, 40 cycles of 95°C for 15 s, 55°C for 20 s, and 72°C for 20 s, with a final melting at 95°C for 20 s. The values of the target genes and the housekeeping gene, *GAPDH*, were calculated for each sample using a standard curve. The standard curve for each gene was constructed from three-fold serial dilutions of a single cDNA sample from an untreated control rat, and the crossing points (CPs) were plotted against an arbitrary *log* concentration of each dilution (in arbitrary units) using Light Cycler 480 Relative Quantification Software. The target genes were then normalized to *GAPDH* within each sample.

**Table 1:** Primer sequences used for qRT-PCR.

Gene symbol	Gene description		Sequence (5'⟶3')	GenBank Accession No.
***GPx*1**	Glutathione peroxidase 1	F:	AAGGTGCTGCTCATTGAGAATG	NM_030826.3
		R:	CGTCTGGACCTACCAGGAACT	
***CAT***	Catalase	F:	ACGAGATGGCACACTTTGACAG	NM_012520.2
		R:	TGGGTTTCTCTTCTGGCTATGG	
***PON*1**	Paraoxonase 1	F:	TGCTGGCTCACAAGATTCAC	NM_032077.1
		R:	TCAAAGCTGAGGACCTTCAAT	
***GAPDH*** *	Glyceraldehyde-3-phosphate dehydrogenase	F:	GGTGAAGTTCGGAGTCAACGGA	NM_017008.4
		R:	GAGGGATCTCGCTCCTGGAAGA	

* housekeeping gene.

### DNA fragmentation and agarose gel electrophoresis

DNA was isolated from hepatic tissue following the method of Kuo, Jan, Jeng and Chiu [39]. The tissue was homogenized in 1 ml lysis buffer [20 mM Tris-Cl (pH 7.5), 0.15 M NaCl, 1 mM EDTA, 1 mM EGTA, 1% Triton X-100, and 25 mM disodium pyrophosphate] at 37°C for 1 h. Then, 0.4 ml of saturated NaCl was added to each set of cell lysates and were incubated on ice for 5 min and centrifuged at 3,000 ×*g* for 30 min. The DNA was precipitated using chilled ethanol, which was separated by centrifugation. Separated DNA was re-suspended in TAE buffer (40 mM Tris-acetate and 1 mM EDTA), which then was electrophoresed on a 1% agarose gel containing 0.5 ug/ml ethidium bromide. The DNA bands were observed and photographed under a UV trans-illuminator.

### Statistical analysis

All data are expressed as mean ± SD. Statistical analysis was carried out using SPSS version 22.0 for Windows (IBM, Armonk, NY, USA). Group differences were analyzed by one-way analysis of variance (ANOVA), followed by Duncan’s multiple range tests; *p* < 0.05 was considered significant.

## Results

### Phytochemical investigation

CE used in this study was characterized with reference to the total phenolic content. The extract was found to be rich in phenols (201 mg gallic acid equivalent/g dry plant material). Moreover, the phytochemical analysis revealed the presence of the following important chemicals: alkaloids, flavonoids, tannins, saponins, anthraquinones, steroids and terpenoids.

### Liver tissue lipid peroxidation and antioxidants status

Compared with untreated controls, rats treated with CCl_4_ alone showed significantly (*p* < 0.05) increased levels of MDA (131%), an indicator of lipid peroxidation, decreased levels of the antioxidant GSH (64%), and decreased activity of the antioxidant enzymes GST (78%), GPx (65%), GR (69%), CAT (69%), PON1 (33%), and AE (64%). In contrast, rats treated with CE alone showed significantly (*p* < 0.05) decreased levels of MDA (90%), increased levels of GSH (113%), and increased activity of GST (107%), GPx (107%), GR (101%), CAT (104%), PON1 (106%), and AE (101%) (Table 2). Compared to rats treated with CCl_4_ alone, those pretreated with CE before CCl_4_ intoxication showed significantly (*p* < 0.05) decreased levels of MDA (90%), increased levels of GSH (135%), and increased activity of GST (123%), GPx (125%), GR (127%), CAT (113%), PON1 (218%), and AE (132%); however, these levels did reach those of the control group (Table 2).

**Table 2:** Effect of aqueous extract of chicory root on the lipid peroxidation biomarker malondialdehyde and antioxidant molecules in the liver homogenates of rats exposed to carbon tetrachloride.

Groups	MDA (nmol/g tissue)	GSH (μmol/g tissue)	GST (U/mg protein)	GPx (U/mg protein)	GR (U/mg protein)	CAT (U/mg protein)	PON1 (U/mg protein)	AE (U/mg protein)
**Control**	77.34 ± 2.45^*c*^	34.12 ± 1.11^*a*^	46.23 ± 3.65^*a*^	22.65 ± 1.98^*a*^	98.34 ± 16.67^*a*^	342.45 ± 43.87^*a*^	33 ± 2.09^*a*^	6760 ± 4.33^*a*^
**CE**	69.98 ± 1.97^*c*^	38.87 ± 1.98^*a*^	49.54 ± 3.23^*a*^	24.28 ± 2.01^*a*^	99.34 ± 11.76^*a*^	354.91 ± 41.75^*a*^	35 ± 2.50^*a*^	6834 ± 4.33^*a*^
**CCl**_**4**_	101.43 ± 3.12^*a*^	21.87 ± 1.87^*c*^	32.11 ± 2.76^*c*^	14.72 ± 1.03^*c*^	67.97 ± 16.78^*c*^	267.34 ± 38.11^*c*^	11 ± 1.13^*c*^	4340 ± 4.33^*c*^
**CE+CCl**_**4**_	91.75 ± 3.56^*b*^	29.56 ± 1.45^*b*^	39.34 ± 3.89^*b*^	18.34 ± 2.02^*b*^	86.23 ± 15.67^*b*^	301.83 ± 37.34^*b*^	24 ± 3.21^*b*^	5750 ± 4.33^*b*^

^(*a*, *b*, *c*)^ Different superscript letters within a column indicate significantly different mean values (*p* < 0.05). CCl_4_, carbon tetrachloride; CE, chicory extract; MDA, malondialdehyde; GSH, reduced glutathione; GST, glutathione S-transferase; GPx, glutathione peroxidase; GR, glutathione reductase; CAT, catalase; PON1, paraoxonase 1; AE, arylesterase.

### Quantitative analysis of hepatic gene expression

To clarify the observed changes in the activities of the antioxidant enzymes, the relative gene expression profiles of some of them in the liver were examined by RT-qPCR. As shown in Table 3, the relative mRNA expression levels of *GPx*1 (21%), *CAT* (22%) and *PON*1 (17%) antioxidant genes were markedly downregulated in the CCl_4_-intoxicated group when compared with the control animals. The expression transcript levels of the target genes were highly significantly upregulated in CE-treated rats in relation to control animals and were additionally significantly upregulated in CE+CCl_4_-treated rats in relation to the CCl_4_-treated group; however, although increased, the expression levels in CE+CCl_4_-treated rats did not reach those of the control animals. As shown in Tables 2 and 3, the changes in the activities of the antioxidant enzymes and the relative expression of their genes are commonly in a positive correlation.

**Table 3:** Effect of aqueous extract of chicory root on mRNA expression levels of antioxidant enzyme genes *GPx1*, *CAT*, and *PON1* in the liver of rats exposed to carbon tetrachloride.

Groups	*GPx*1	*CAT*	*PON*1
**Control**	4.54 ± 0.73^*a*^	3.43 ± 0.73^*a*^	4.35±0.62^*b*^
**CE**	6.54 ± 0.49^*a*^	4.12 ± 0.44^*a*^	5.35±0.34^*a*^
**CCl**_**4**_	0.96 ± 0.33^*c*^	0.76 ± 0.41^*c*^	0.75±0.34^*d*^
**CE+CCl**_**4**_	3.50 ± 0.63^*b*^	1.87 ± 0.53^*b*^	2.62±0.63^*c*^

^(*a*, *b*, *c*, *d*)^ Different superscript letters within a column indicate significantly different mean values (*p* < 0.05). CCl_4,_ carbon tetrachloride; CE, chicory extract; *GPx*1, glutathione peroxidase 1; *CAT*, catalase; *PON*1, paraoxonase 1.

### Electrophoretic pattern of DNA fragmentation

As shown in Fig. 1, agarose gel electrophoresis of the DNA confirmed the results of the colorimetric assays of lipid peroxidation, antioxidant status, and corroborated the changed levels of the gene transcripts. The liver samples of CCl_4_-intoxicated rats showed smeared DNA fragmentation, as evident from the tailing of the DNA (Lanes 5–9) when compared with the control (Lanes 1 and 2) and the CE-treated (Lanes 3 and 4) groups. Pretreatment of CCl_4_-intoxicated rats with CE markedly suppressed DNA fragmentation (Lane 10), where DNA was still localized at the starting point. There was no significant difference between the DNA electrophoretic patterns of the CE-treated rats and the control groups.

**Fig 1:** Agarose gel electrophoresis of extracted DNA from liver of rats. Results of the DNA fragmentation assay confirm that pretreatment with chicory extract attenuates CCl4-induced hepatotoxicity in rats. Lane M, DNA ladder; Lanes 1–2, untreated control group; Lanes 3–4, chicory extract-treated group; Lanes 5–9, CCl4-treated group, and Lane 10, chicory extract+CCl4-treated group.

## Discussion

Severe hepatic injuries caused by toxic chemicals, drugs, and infections can be difficult to manage; however, plant extracts have shown promise in treating hepatic failure due to severe oxidative stress [10, 40]. Oxidative stress occurs when the balance between ROS and antioxidants is disrupted, resulting in the dysregulation of cellular functions and leading to various pathological conditions [41]. Elevated levels of MDA (end product of LPO) and decreased levels of GSH (primary redox regulator) are important indicators of oxidative stress [5]. Our results show that pretreatment with CE attenuates CCl_4_-induced changes in MDA and GSH levels in rats, suggesting free radical scavenging properties. The antioxidant GSH directly scavenges ROS and free radicals, or being a part of the GSH redox system; GPx, GR and GST [41, 42], thereby protecting biological systems from oxidative stress. CAT is a heme protein that catalyzes the reduction of H_2_O_2_ to water and oxygen, thereby protecting cells from highly reactive hydroxyl radicals [43]. Similarly, the selenoenzyme GPx plays an important role in the reduction of H_2_O_2_ and hydroperoxides. The enzyme GST catalyzes the conjugation of GSH with electrophilic xenobiotics, and GR utilizes NADPH to reduce GSH [44]. Previous studies have also reported that the CCl_4_ decreases the activity of enzymes in the GSH redox system in the liver, implicating its role in the pathogenesis of hepatotoxicity [7, 40, 45]. Moreover, the results of our study were consistent with previous studies reporting that the hepatoprotective activity of CE is mediated through increased activity of enzymatic and non-enzymatic antioxidants [21, 46–50]. The protective effect of CE against CCl_4_-induced hepatic oxidative damage may be due to the presence of antioxidant compounds such as anthocyanins, flavonoids, polyphenols, and vitamin C [51, 52]. The phytochemical screening of CE confirmed the presence of such bioactive compounds, particularly total phenolics, which may contribute to protection of CE against free radical generation and hepatotoxic effects of CCl_4_.

PON1 and AE are high-density lipoprotein (HDL)–associated enzymes synthesized in the liver, which are potential antioxidants [53]. The activity of these enzymes may be particularly meaningful as an index of liver function and for monitoring chronic hepatitis [54]. Exogenous and endogenous oxidant agents readily inactivate PON1 and AE [55], thereby decreased activity of PON1 and AE is strongly associated with the development of oxidative liver damage [56–58]. In our study, the increased hepatic PON1 and AE activities in rats pretreated with CE before CCl_4_ intoxication appears to be due to natural antioxidants present in chicory roots. Previous studies have shown that PNO1 and AE activities can be induced by polyphenols [59, 60], flavonoids [61], and vitamin C and E intakes [62]. PON1 and AE enzymes metabolize toxic oxidized lipids of low-density lipoprotein (LDLs) and HDLs [53], their increased activities may underpin the remarkable antioxidant effect of CE on LDL and its inhibitory effect on the production of thiobarbituric acid-reactive substances and the degradation of the LDL fatty acids [23], thereby protecting against CCl_4_-induced oxidative damage.

The liver expression profiles of genes encoding antioxidant enzymes-associated with HDLs (*GPx*1, *CAT*, and *PON*1) were investigated to provide insight into the mechanisms governing their activities. Microarray studies have described changes in gene expression caused by CCl_4_ toxicity [63, 64], revealing molecular responses to CCl_4_ and the genetic basis of hepatotoxicity. The low activity of antioxidant enzymes in liver tissue caused by CCl_4_ toxicity appears to be a result of not only oxidative tissue damage but also to altered enzyme structure, function, and expression [7]. Oxidative stress in liver tissue caused by CCl_4_ intoxication may lead to inactivation of GPx, CAT, and PON1, or reactive intermediates of CCl_4_ bioactivation may bind to these enzymes [65, 66]. Consistent with the CCl_4_-induced changes in antioxidant enzyme activity and expression observed in the present study, Manubolu et al. reported that altered patterns of enzyme activity during oxidative stress are due to a shift in gene expression [65]. Supplementation with exogenous antioxidants during periods of increased oxidative stress appears to increase activity of the antioxidant defense system by stimulating synthesis of antioxidant enzymes [67]. In this study, supplementation with CE appeared to boost antioxidant enzyme activities by upregulating gene expression. The overexpression of genes encoding antioxidant enzymes thus provides strong protection against the development of experimental liver disease [68]. Results of the DNA fragmentation assay confirmed the proteins, enzymes and gene expression findings, indicating that the CE is able to inhibit CCl_4_-induced DNA damage [46], and further the hepatotoxicity directly by removing ROS.

Taken together, our results show that the hepatoprotective effect of *C*. *intybus* L. is likely due to the prevention of LPO, sustaining of endogenous antioxidant molecules, and overexpression of genes encoding antioxidant enzymes, thereby preventing DNA damage. This effect appears to be mediated by natural antioxidants in chicory roots, which significantly attenuated the oxidative threat and led to normal hepatic functions. Further research must be conducted to elucidate the mechanisms regarding the hepatoprotective effect of CE at the molecular level.
